# Molecular modeling of the structural, electronic, excited state dynamic, and the photovoltaic properties of the oligomers of n-corannulene (n = 1–4)

This article has been retracted.

**DOI:** 10.1016/j.heliyon.2023.e20706

**Published:** 2023-10-06

**Authors:** Hamid Hadi, Hitler Louis, Terkumbur E. Gber, Festus O. Ogungbemiro

**Affiliations:** a Department of Chemistry, Physical Chemistry group, Lorestan University, Khorramabad, Iran; b Computational and Bio-Simulation Research Group, University of Calabar, Calabar, Nigeria; c Centre for Herbal Pharmacology and Environmental Sustainability, Chettinad Hospital and Research Institute, Chettinad Academy of Research and Education, Kelambakkam 603103, Tamil Nadu, India

**Keywords:** n-Corannulene, Molecular design, Excitation, Photovoltaic properties

## Abstract

Despite the fact that n-corannulene oligomers (n = 1–4) have a variety of electronic and optical properties, including the ability to be tuned and the potential to be used as light-harvesting materials, there has not been a computational assessment of their structural, electronic, and optical properties. Herein, a computational evaluation of the concerned materials regarding their potent use in solar cell technology has been conducted via DFT/CAM-B3LYP and M062X/6-311+G level of theory. It was observed that the calculated 1st frequency of the n-Corannulene (n = 1–4) were 144.15, 106.36, 48.96 and 42.21 respectively. Notably, the computed cohesive energy value increased as the number of Corannulene units increases while the electronic characteristics revealed that the chemical activity of the structures increased as the number of oligomers rose. Both calculation techniques demonstrate that the number of n-Corannulene oligomers increases the HOMO energy while decreasing the LUMO energy based on the external electric field (EF) effect. The findings demonstrated that as EF intensity increases, the energy gap (Eg/eV = |E_HOMO_-E_LUMO|_) of these molecular systems decreases which can be attributed to a decrease in the electron transfer potential barrier. The 4-Corannulene systems showed the highest wave length of adsorption for the investigated compound at 546.18 nm, with the highest oscillator strength of 0.2708 and the lowest transition energy of 2.2700 eV, arising from S0–S1 (H-L) and the highest major percentage contribution of 93.34 % in comparison to the investigated compounds. We are hopeful that this research will help experimental researchers understand the potential of n-Corannulene, specifically 4-corannulene, as powerful material for a variety of applications ranging from solar cell, photovoltaic properties and many others.

## 1 Introduction

More than 30 years ago, Barth and Lawton created corannulene, which has a distinctive design in the form of a bowl [1,2]. One of the first instances of the entire sp2 carbon network being curved [3]. The properties of this intriguing material have been subject to previous studies. Corannulene, classified as an unsaturated hydrocarbon, is composed of fused rings, featuring a central five-membered ring and five peripheral six-membered rings [[4], [5]]. Its composition bears resemblance to C_60_, but differs significantly in structure. Corannulene exhibits a curved p surface, distinguishing itself from C_60_ by featuring two distinct faces: a concave interior and a convex exterior.". Corannulene is an extremely symmetric compound (C5V) in the polycyclic aromatic hydrocarbon family. Graphene, a limiting zero-curvature instance, is one of the most hopeful compounds in nanotechnology. Non-hexagonal bands, such as fullerenes, have been shown to cause non-zero curvature in graphene sheets. Corannulene is comparable to defective graphene in that one of its hexagons has been substituted with a pentagon [[6], [7]]. Due to the destabilization of pi electrons, it emerged that oligomers made of Corannulene molecules have outstanding electrical and optical characteristics. Scientists have been researching hard to improve the properties of these materials and develop novel nanomaterials.

In recent years, the rapid advancements in technology have led to the widespread adoption of computational (DFT) software by numerous research groups. This powerful tool finds applications in various fields, including nanosensors, evaluation of electrical and optical properties, drug development, and biosensors [[8], [9], [10]]. Notably [11], explored the geometric and electrical structures of regular and doped ethylene dioxythiophene (EDOT) oligomers using density functional theory and Hartree-Fock methods. Additionally, they reported semiempirical optical properties based on shapes obtained from DFT and HF (intermediate disregard of differential overlap/single configuration, (INDO/SCI)). Similarly, Zade [12], extensively investigated a wide range of materials, from short conjugated oligomers to conjugated polymers. Through their research on long conjugated oligomers and the inclusion of counterions in oligothiophenes and polymers with repetitive polar units, they gained valuable insights. They emphasized that different properties manifest in various ways and, to accurately infer polymer properties, lengthy oligomers (with approximately 50 double bonds in the backbone) are often required. Utilizing DFT, Jarmelo [13] conducted experimental (IR/Raman and 1H/13C NMR) and theoretical (DFT) studies on the special conformations adopted by l-lactic acid oligomers and poly (l-lactic acid) homopolymer. They successfully characterized the preferred conformations adopted by PLLA chains by comparing calculated energies and computed vibrational and NMR spectra of the most stable conformers with experimental data.

### 1.1 Top of form

In spite of such attempts, few or no works on the design and numerical assessment of structural, electronic, and optical characteristics of n-Corannulene (n = 1–4) oligomers have been discovered. As a result, the Molecular modeling of the structural, electronic, excited state dynamic, and the photovoltaic properties of the oligomers of n-Corannulene (n = 1–4)" is investigated herein using (DFT/CAM-B3LYP/6-311+G and DFT/M062X/6-311+G) to deepen our understand on the behavior and properties of a specific class of molecules called oligomers of n-Corannulene such as molecular structure, electronic properties, excited state dynamics, and photovoltaic (solar cell) properties of these oligomers. We employed UV excitation analysis to study the behavior of the oligomers upon excitation, including the relaxation processes, electronic transitions, and excited state lifetimes. This analysis provides insights into the excited state behavior and potential for light-harvesting applications. Similarly, the Photovoltaic Properties evaluation was performed on the photovoltaic properties of the oligomers, including their absorption spectra, charge transport properties, and potential for solar energy conversion. This analysis helps assess the suitability of the oligomers for use in photovoltaic devices such as solar cells.

## 2 Computational details

The modelled structures were sketched using Gaussveiw 6.0.16 [14] and all theoretical calculations were achieved with the help of Gaussian (G09) suit of programs software [15] To embark on our scientific journey, we harnessed the power CAM-B3LYP (short for Coulomb-attenuating method with B3LYP functional): CAM-B3LYP and M062X are two powerful hybrid functional methods commonly used in Density Functional Theory (DFT) calculations. CAM-B3LYP combines the Becke three-parameter exchange functional (B3) with the Lee-Yang-Parr correlation functional (LYP), while M062X combines the Minnesota functional (M06) with the Becke exchange functional (X) [16]. In this study, these theoretical methods were employed in conjunction with the reliable 6-311+G basis set for the structural equilibration [16]. These functionals were chosen due to their well-documented and superior performance in calculating reaction energies, barrier heights, and transition states, particularly for organic and inorganic reactions in photovoltaic applications [17]. Consequently, they have demonstrated their reliability and effectiveness in similar contexts. For the examination of the designed structures' feasibility, two critical parameters were investigated: vibration frequency and cohesive energy (as represented by Equation (1)). These parameters play a crucial role in evaluating the potential success of each intended structural design [18]**.**

(1) $$E_{Coh}=-(E_{tot}-\sum_{i}n_{i}E_{i})/n$$

Where E_tot_, E_i_, and n_i_ are the total energy of all designed molecules, the atomic energy and the number of atoms respectively and n is the total number of all atoms. The key factor that determines the intrinsic properties of all types of molecules is the position of the conduction and valence bands and the gap between them. The density of electronic state (DOS) and energy gap (Equation (2)) were checked to check the electronic properties of each of the designed structures using the GaussSum03 software [19].

(2) Eg/eV=|ELUMO−EHOMO|

E_HOMO_ denotes the energy of the highest filled molecule orbital (HOMO), while E_LUMO_ denotes the energy of the lowest unoccupied molecular orbital. (LUMO). In addition, the electron density map of each proposed structure was assessed using the Multiwfn program [20]. The UV–visible absorption spectrum of each of the designed structures was computed from the optimized geometry using CAM-B3LYP and M062X method and 6-311+G basis set using time-dependent density functional theory (TD-DFT). Radiant lifetime and light harvesting efficiency (LHE) were investigated in order to investigate the photovoltaic properties of each of the designed structures (Equation (3), (4))).

The radiative lifetimes (in au) for spontaneous emission were calculated using the Einstein transition probability using the method 3 [21].

(3) τ=C32(EFlu)2f

Where (c) = velocity of light, E_Flu_ = the excitation energy, and = oscillator strength (O.S.) [22].

The LHE parameter is related to the oscillator strength (f).

(4) $$LHE=1-10^{-f}$$

f is the oscillator strength in the complex, which corresponds to the λmax.

Finally, in order to investigate the possibility of using each of the designed structures in molecular nanoelectronic systems, the effect of different electric fields on each of the structures was investigated. For this purpose, the electrical conductivity (G) of each of the designed structures was obtained using the Landauer-Boettiker formula (Equations (4), (5), (6))).

(4a) $$G=\frac{1}{R}=\frac{2e^{2}\tau_{e}}{\hbar }$$

(5) τ=exp(−βL)

(6) $$\beta ={\left(\frac{2m^{*}\alpha \varphi }{\hbar^{2}}\right)}^{\frac{1}{2}}$$

where ℏ is $\frac{h}{2\pi }$, φ is the potential barrier height for tunneling through the HOMO or LUMO level, equal to the energy differential between the Fermi energy and the molecule HOMO or LUMO level, in this symmetric situation, m* is the effective mass of the electron (m* = 0.16m0, m0 is the free electron mass) and is the symmetry component in the potential profile. α = 1 [[23], [24], [25]].

## 3 Results and discussion

### 3.1 Molecular design and geometric structures

Geometry optimization of Corannulene and its oligomers structure with 2–4 units was performed to generate a more stable structures as presented in Fig. 1, using hybrid CAM-B3LYP function in conjunction with 6-311+G basis sets. First imaginary frequency and cohesive energy per carbon atom were examined as fundamental variables in the stability of constructed structures. (Table 1). The calculated first frequencies of the n-Corannulene (n = 1–4) were 144.15, 106.36, 48.96, and 42.21, indicating that all frequencies are positive and can be a significant cause for the stability of the proposed structures [26]. To evaluate the comparative stability of the investigated structures, their energy values were computed using the CAM-B3LYP and M062X computational levels along with the 6-311+G basis set. An interesting observation is that the cohesive energy value increases with the number of Corannulene units, suggesting a notable inclination of Corannulene to polymerize and form oligomers. Table 1 displays the computed values of cohesive energy acquired using two different techniques. The presence of imaginary frequency and the high cohesive energy indicate the potential of creating planned structures [27,28]. It is important to know that upon comparing the obtained geometry parameters like bond length with the experimental results of Anil et al. [29] in literature, a strong correlation was observed. From the geometry of n-Corannulene (n = 1) the C8 – C13 (1.42 Å), C7 – C8 (1.42), C18–C9 and C12 – C14 had 1.45 Å respectively. Similarly, the five-member ring of the studied structured was observed with a bond length of C3 – C4 and C13 – C12 of 1.39 correlating perfectly well with the previously reported works.

**Fig. 1:** Optimized structure and IR spectrum of each designed structure (a = n-Corannulene (n = 1), b = n-Corannulene (n = 2), c = n-Corannulene (n = 3), and d = n-Corannulene (n = 4), respectively obtained at (CAM-B3LYP/6-311+G).

**Table 1:** The obtained results reveal the cohesive energy values within the designed structures.

Structure	Cohesive energy (Kcal.mol^−1^) (CAM-B3LYP)/6-311+G	Cohesive energy (Kcal.mol^−1^) (M062X)/6-311+G
**Corannulene**	132.30	133.05
**2- Corannulene**	156.34	155.98
**3- Corannulene**	184.75	184.01
**4- Corannulen**	214.83	213.96

The analysis of the IR spectrum of each of the suggested structures, on the other hand, revealed that the first IR frequency is positive for all of the designed structures, indicating that these structures are not in a transition state. (Fig. 1). The lack of imaginary frequency and cohesive energy computations guaranteed the safety of the planned structures.

### 3.2 Electronic properties

Understanding electronic structures is crucial for interpreting absorption bands. Fig. 2, Fig. 3 display the estimated energies of the frontier orbitals HOMO and LUMO, as well as the energy gaps (Eg/eV). Additionally, the DOS spectra, determined using the CAM-B3LYP/6-311+G and M062X/6-311+G methods, are available in the supplemental data [30,31]. The HOMO represents the valence band, while the LUMO corresponds to the conduction band of molecules. Analyzing the energy levels of these orbitals provides valuable insights into molecular activity.

**Fig. 2:** Presents the Iso-surface of the frontier orbitals, HOMO and LUMO, along with their corresponding energy gaps for the studied Corannulene structures (n = 1–4) obtained using the CAM-B3LYP and M06-2X methods.

**Fig. 3:** **3(a)**The energy effect of HOMO and LUMO frontier orbitals on the energy gap (Eg/eV) of each of the designed structures (CAM-B3LYP method)**. 3(b) T**he process of changing the energy gap of each of the designed structures by increasing the number of oligomers.

In general, negative LUMO energy levels suggest strong chemical activity of the structures, so E_LUMO_ gives an approximation of electron affinity (A = -E_LUMO_) [[32], [33], [34], [35]]**.** Similarly, E_HOMO_ can estimate the ionization potential (I = -E_HOMO_). As a consequence, the E_LUMO_ values strongly suggest that more chemically active species are created as a result of structure hybridization. This is also true for the ionization energy determined from E_HOMO_, and it has been demonstrated that the ionization energy of each of the designed structures diminishes as a consequence of their development. Therefore, the chemical activity of the structures increases with the increase in the number of oligomers. According to the results obtained from the NBO analysis, 4-Corannulene showed the highest chemical activity. This feature shows that 4-Corannulene can be used in targeted molecule.

The findings of both calculations indicate that increasing the number of n-Corannulene oligomers increases the HOMO energy while decreasing the LUMO energy. when the n-Corannulene oligomers are exposed to electron-donating species or in a reducing environment, the oligomers will readily accept electrons due to their low LUMO energy. As a result, the oligomers may undergo reduction reactions, where the addition of electrons can lead to the formation of larger oligomers with a higher number of corannulene units. On the other hand, if the LUMO energy level is relatively high, the molecule has a lower electron affinity and is less likely to accept electrons. In the case of n-Corannulene oligomers, a high LUMO energy would indicate a reduced propensity to accept electrons [36,37]. Consequently, a remarkable 49.5 % decrease in the energy gap is observed in 4-Corannulene. Notably, the comparison between the energy of HOMO and LUMO frontier orbitals and the energy gap highlights the significant influence of the LUMO frontier orbital on this gap [34,35]. By reducing the energy gap in the molecule, the possibility of quantum tunneling arises, potentially enhancing the electrical conductivity of the examined structure. The amplified electrical conductivity of oligomers, with an increasing number of units, can be attributed to the elongation of the π-electron chain or an increase in hyper-conjugation among these electrons. This characteristic designates 4-Corannulene as a potential component in molecular nanoelectronic systems. Further details on this topic will be expounded upon in subsequent sections.

### 3.3 Dipole moment and electronic spatial extent (ESE)

The dipole moment was investigated as one of the effective parameters in solubility (Fig. 4). Compounds with greater dipole moments are more soluble in polar liquids such as water. The results showed that with the increase in the number of oligomers, the dipole moment and the spatial extent of the electron increase significantly. The cause of such an issue may be attributed to the growth of the conjugated foot bond in each of the proposed structures [38,39]. Table 1 shows that the dipole moment of Corannulene is very low, and its solubility in water is very low. As a result, if this structure is used as a base substance in the production of electrochemical sensors, it can have a lengthy life. Because most electrochemical sensors, such as ion-selective electrodes, lose their sensitivity over time due to sensor material leaking into solutions.

**Fig. 4:** Dipole moment and Electronic spatial extent for designed structures.

### 3.4 Electrostatic potential (ESE) and electron density map

The molecular electrostatic potential offers valuable insights into various characteristics, including molecular size, dipole moment, structure, electronic density, hydrogen bonding interactions, and chemical reactivity [40]. In this representation, red indicates electron-rich regions (partially negative charge), while yellow represents electron-poor areas (partially positive charge). Fig. 5 displays the electrostatic potential map for the subject molecule, studied using the CAM-B3LYP/6-311+G (d,p) technique. The red (electron-rich) area is found at the lateral edges of the structure, where electrophilic attack is feasible. The findings indicate that increasing the number of Corannulene units raises the electron density at both the structure's borders and its core. The expansion of π-bonds in the structure causes a rise in electron density. In Fig. 5 (Left), the bonding regions of C–C and C–H bonds are readily identifiable. However, it's important to note that the small white circles in the carbon aromatic ring centers do not correspond to 1s electrons. Instead, they arise from the penetration effect of valence atomic orbitals into the core region.

**Fig. 5:** presents the electron density map (left) and the electrostatic potential (ESP) map (right) for the designed structures. (a = n-Corannulene (n = 1), b = n-Corannulene (n = 2), c = n-Corannulene (n = 3), and d = n-Corannulene (n = 4), respectively.

### 3.5 Optical properties

In order to explore the optical properties of the designed structures, their UV–Visible spectra were calculated using the TD-DFT method at the CAM-B3LYP/6-311+G and M062X/6-311+G levels. The results of these calculations, illustrating the UV–Visible spectrum of the designed structures, are presented in Fig. 6.

**Fig. 6:** displays the adsorption intensity and corresponding wavelengths for the studied Corannulene structures (n = 1–4) as a function of wavelengths obtained using the CAM-B3LYP and M062X methods.

In order to comprehend the optical characteristics of the designed molecules, the UV–Visible light absorption was quantified using the TDDFT technique. Fig. 6 illustrates a comparison of the UV–Visible absorption measurements obtained for the proposed structures. To ensure data accuracy, calculations were performed using the CAM-B3LYP and M062X methods. Notably, 4-Corannulene exhibited higher optical activity compared to the other compounds, as evidenced by the statistics presented in Fig. 6. This structure exhibits one significant absorption in the visible region, suggesting that it is more optically active than the other structures. In reality, increasing the amount of Corannulene units enhanced the optical properties considerably [41,42]. This was anticipated as a result of the increased length of the π-bond conjugated structure and decreased energy gaps. One of the variables influencing photocurrent density is the energy gap. Differences, in energy gaps in general, make electrons more readily excited, which is advantageous for capturing longer-wavelength light. However, as the number of corannulene oligomers increases, the energy gap of the molecules progressively diminishes, suggesting that increasing the number of oligomers is very helpful in moving the absorption bands to the longer wavelength. This characteristic causes more photons to be absorbed in a given period in a solar cell, which may increase short circuit current density JSC and power conversion efficiency. (η).

### 3.6 External electric field effect

In order to check electrical conductivity, each of the designed structures was subjected to electric field (EF in +X) with different intensities [[43], [44]] and the proposed structures in exchange for the external electric field effect (+X) is presented in Table 2. For this purpose, the effects of EF on HOMO/LUMO frontier orbitals and the length of each molecular system were investigated (Table 3 and Fig. 7). The findings demonstrated a noticeable decrease in the energy gap (Eg/eV = |E_HOMO_-E_LUMO_|) of these molecular systems with increasing EF intensity. This reduction in the energy gap can be attributed to the decreased electron transfer potential barrier. Furthermore, the impact of the external electric field (EF) on the length of these molecular systems (n-Corannulene) revealed a reduction in the length of each structure as the electric field's intensity increased [45,46]. The EF effects on length of the organic molecular systems can be because of the positive and negative charge centers separation and as well as reducing dihedral and tetrahedral angles in these systems, as structure responses to applied external EF (see Table 4).

**Table 2:** HOMO/LUMO frontier orbitals changes, Eg/eV and also the length of each of the proposed structures in exchange for the external electric field effect (+X).

Corannulene					2-Corannulene			
Field (10^−4^ a.u)	**LUMO (eV)**	**HOMO (eV)**	**Eg/eV (eV)**	**Length (A)**	**LUMO (eV)**	**HOMO (eV)**	**Eg/eV (eV)**	**Length (A)**
0	−1.58	−6.02	4.44	6.5259	−2.3	−5.56	3.26	12.3702
20	−1.91	−6.29	4.38	6.5199	−2.32	−5.55	3.23	12.3670
40	−1.59	−5.98	4.34	6.5197	−2.39	−5.53	3.14	12.3648
60	−1.61	−5.94	4.33	6.5182	−2.49	−5.44	2.95	12.3631
80	−1.64	−5.9	4.26	6.5154	−2.61	−5.27	2.66	12.3621
100	−1.68	−5.86	4.18	6.5148	−2.75	−5.09	2.34	12.3613
3-Corannulene					**4-Corannulene**			
Field (10^−4^ a.u)	**LUMO (eV)**	**HOMO (eV)**	**Eg/eV (eV)**	**Length (A)**	**LUMO (eV)**	**HOMO (eV)**	**Eg/eV (eV)**	**Length (A)**
0	−2.52	−5.46	2.94	14.7845	−2.99	−5.19	2.20	17.4288
20	−2.55	−5.44	2.89	14.7786	−3.0	−5.18	2.18	17.4199
40	−2.63	−5.38	2.75	14.7753	−3.04	−5.16	2.12	17.4161
60	−2.72	−5.31	2.59	14.7733	−3.1	−5.11	2.01	17.4138
80	−2.83	−5.22	2.39	14.7720	−3.18	−5.05	1.87	17.4120
100	−2.95	−5.11	2.16	14.7699	−3.28	−4.98	1.70	17.4102

**Table 3:** The global quantum descriptors parameters for the studied compounds (Corannulene, 2-Corannulene, 3-Corannulene and 4-Corannulene) all calculated in (eV).

Compounds	Band gap	IP	EA	Σ	η	μ	ω	χ
Corannulene	4.4412	6.0181	1.5769	0.2252	2.2206	−3.7975	3.2471	3.7975
2-Corannulene	3.2610	5.5560	2.2986	0.3067	1.6305	−3.9290	4.7340	3.9290
3-Corannulene	2.9413	5.4597	2.5184	0.3399	1.4706	−3.9890	5.4101	3.9890
4-Corannulene	2.2047	5.1947	2.9899	0.4536	1.1023	−4.0923	7.5962	4.0923

**Table 4:** Transition types, absorption energy, Wavelength, Oscillator strength, Major contribution and Transition of the studied systems (Corannulene, 2-Corannulene, 3-Corannulene and 4-Corannulene).

Systems	Transition Type	Energy/eV	Wavelength (nm)	Oscillator strength (*f*)	Percentage contribution	Transition
**Corannulene**	S_0_→ S_1_	3.9711	312.22	0.0000	65 -> 66(48.94)	H → L
**2-Corannulene**	S_0_→ S_1_	3.3607	368.92	0.0000	114 ->116(81.93)	H-1 → L
**3-Corannulene**	S_0_→ S_1_	2.9913	414.49	0.0184	163 ->165(76.89)	H-1 → L
**4-Corannulene**	S_0_→ S_1_	2.2700	546.18	0.2708	200 -> 201(93.34)	H → L

**Fig. 7:** Graph of changes in energy gap and length of the structure in response to the application of an external electric field. (a = n-Corannulene (n = 1), b = n-Corannulene (n = 2), c = n-Corannulene (n = 3), and d = n-Corannulene (n = 4), respectively.

### 3.7 Global quantum descriptors

To unravel details information about the studied compounds stability and reactivity, we summoned the ingenious Koopman's approximation, invoking its power to calculate the global chemical reactivity indices. Excitingly, we witnessed the revelation of essential quantum reactivity indices, including the enigmatic chemical potential (μ), the chemical hardness (η), the delicate chemical softness (σ), the electronegativity index (χ), and the electrophilicity index (ω). Employing the highly effective Koopman's approximation, which establishes a connection between the energies of the HOMO and LUMO to the Ionization Potential and the Electron Affinity respectively, we calculated the results of the global quantum reactivity indices displayed in Table 3, following the equations outlined in the literature. (7- 12).

(7) $$\text{IP}={-E}_{\text{HOMO}}$$

(8) $$\text{EA}={-E}_{\text{LUMO}}$$

Therefore, utilizing the provided equations, we can compute the global reactivity descriptors. (9)–(12) [38].

(9) $$\chi =-\mu =\frac{IP+EA}{2}$$

(10) η=12(IP−EA)=ELUMO−EHOMO2

(11) $$\omega =\frac{\mu^{2}}{2\eta }$$

(12) $$\sigma =\frac{1}{2\eta }=\frac{1}{2\left(IP-EA\right)}=\frac{1}{E_{\text{LUMO}}-E_{\text{HOMO}}}$$

From the results presented in Tables 3 and it was observed that all the number of chains of Corannulene increases there was a corresponding increase in the softness of the studied structure such that a given pattern was observed as thus, Corannulene < 2-Corannulene < 3-Corannulene < 4-Corannulene with corresponding energies 0.2252 eV, 0.3067 eV 0.3399 eV and 0.4536 eV respectively. The observed range in the chemical softness values reflects the sensitivity of a material's electronic structure to changes in its environment, particularly when exposed to light or electromagnetic radiation which in the context of photovoltaics, the higher chemical softness of 0.4536 eV from 4-Corannulene indicates that the material is more responsive to external stimuli. Similarly, the chemical hardness was observed in the revised case, as the number of Corannulene increases, the chemical hardness values decrease [47,48]. This observation was in agreement with the frontier molecular orbital gap. It is worth knowing that the enigmatic chemical potential (μ), the e electronegativity index (χ), and the electrophilicity index (ω) were also in relation to each other a regard the compounds stability and reactivity. Importantly, higher chemical softness in photovoltaic properties studies is desirable as it signifies a material's enhanced responsiveness to light, resulting in improved photon absorption and efficient charge transport, ultimately leading to higher conversion efficiency in solar cells.

In addition, based on Landauer's theory, the effect of EF (+X) on the current-voltage (I–V) curve of these molecular systems can be observed (Fig. 8). The results show that with the increase in the number of corannulene oligomers, the electrical conductivity increases significantly (the electrical conductivity of 4-Corannulene increased significantly with increasing EF intensity).

**Fig. 8:** Current-voltage diagrams (I–V) of the designed structures (n-Corannulene) studied in this work.

### 3.8 Excited state dynamics

#### 3.8.1 UV-excitation analysis

To design better devices, many electronic devices, such as LEDs, solar cells, and lasers, rely on excitation and relaxation processes to function [49,50]. By studying these processes, designing more efficient and effective devices that utilized these processes to their full potential become important to scientists. To gain more knowledge into the underlying different variation among the excited state in the studied compound's excited-state characteristics, a complete excitation-based analysis is used. This is given that descriptions based on extended pi conjugated systems and molecular orbitals do not always provide a full image [51]**.** The excitonic analysis based on Rather, coupled electron–hole pair present a proficient and appropriate quantitative measure. From the result presented in Table 3 herein, the frank-Condon excitation for the Corannulene was observed from H → L excitation with an excitation energy of 3.9711eV, wavelength of 312.22 nm and a major contribution of 48.94%. From the 2-Corannulene S_0_ → S_1_ transition was observed due to the combination of H-1 → L, this had an excitation energy of 3.3607 eV and 368.92 nm with corresponding 81.93%. The first two systems had the least *f*_*osc*_ values. The first transition in 3-Corannulene shows a major peak appearing at 2.9913 eV (*f*_*osc*_ = 0.0184), with the wavelength of 414.49 nm corresponding to a transition between H-1 → L and a respective contribution of 76.89 %. The highest wave length of adsorption for the studied compound was observed in the 4-Corannulene systems with 546.18 nm having the higher oscillator strength of 0.2708 with the lowest transition energy of 2.2700 eV arising from S_0_ → S_1_ (H → L) with the highest major percentage contribution of 93.34% compared to the studied compounds. This was observed to concur with the least energy gap of the 4-Corannulene compound as compared to its counterpart. Furthermore, due to the various adsorption energy and wavelength of the adsorption spectral, the key configurations involved in the transitions are very unique in all of the research compounds. The ultraviolet analysis shows that the generation of a low-lying excited CTTS state can be initiated by either direct monophotonic absorption in the low energy tail of the CTTS ground state.

#### 3.8.2 Excited state relaxation

The concept of relaxation is very important in various fields, as it relates to the restoration of equilibrium and the reduction of stress and tension, in physics and chemistry, relaxation often refers to the process by which a system returns to a state of equilibrium or stability after being perturbed [52,53]. This can include the relaxation of an excited state of an atom or molecule back to its ground state. In addition, relaxation can refer to the relaxation of magnetic or electric fields in materials, the relaxation of mechanical stresses in solids, or the relaxation of temperature or pressure gradients in fluids. The excited energy relaxation in the studied compounds were investigated in this study and the obtained results are presented in Table 5: From the results, it can be observed that for Corannulene compound the relaxation energy of 3.9710 eV was noticed with wavelength of 312.22 nm, corresponding to a lower oscillator strength and major percentage contribution of 53.17%. This was observed from the 65 -> 66 (H → L). Similarly, the relaxation energy for the 2-Corannulene compound was as observed from the S_0_ → S_1_ type was 3.3607 eV with a wavelength of 368.92 nm. The orbital relaxation was observed from the respective orbital 65 -> 66 (H-1 → L) with a major contribution of (81.93 %). On the other hand, the relaxation energy noticeable in the 3-Corannulene compound observed from S_0_ → S_1_ was 2.9040 eV with relaxation wavelength of 426.94 nm correspond to and oscillator strength of 0.1191. The orbital contribution of the compound was from 164 to >165(H → L) with the major contribution of (79.59 %). Furthermore, the relaxation energy for the 4-Corannulene compound as observed from the S_0_ → S_1_ relaxation type was 2.2700 eV with the highest wavelength of 546.18 nm and an oscillator strength of 0.2710 arising from the 200 -> 201(H → L) orbitals with a corresponding major contribution of (93.33 %). This is important for advancing our understanding of the physical world and developing new technologies and materials with important practical application.

**Table 5:** Relaxation types, relaxation energy, Wavelength, Oscillator strength, Major contribution and Transition of the studied systems (Corannulene, 2-Corannulene, 3-Corannulene and 4-Corannulene).

COMPOUND	Relaxation Type	ENERGY/eV	Wavelength (nm)	Oscillator strength (*f*)	% Contributions	Transition
**Corannulene**	S_0_→ S_1_	3.9710	312.22	0.0000	65 -> 66 (53.17)	H → L
**2-Corannulene**	S_0_→ S_1_	3.3607	368.92	0.0000	114 ->116 (81.93)	H-1 → L
**3-Corannulene**	S_0_→ S_1_	2.9040	426.94	0.1191	164 ->165 (79.59)	H → L
**4-Corannulene**	S_0_→ S_1_	2.2700	546.18	0.2710	200 -> 201 (93.33)	H → L

#### 3.8.3 Photovoltaic properties

The spectral dispersion of sunlight that is absorbed into the molecule is measured by light harvesting effectiveness (LHE). The LHE is an essential property in solar cells and plays a key role in thus increasing short-circuit current density JSC. Furthermore, an increase in Radiant lifespan will slow down the charge recombination process and improve the efficacy of photovoltaic cells, resulting in high light-emitting efficiency [54,55]. The values obtained for LHE and radiative lifetimes with the calculation method (TD-DFT) CAM-B3LYP/6-311+G are shown in Fig. 9. According to the obtained results, with the increase in the number of oligomers, the values of LHE and radiative lifetimes increase (Due to better π conjugation). This light harvesting efficiency plays a crucial role in the study and development of photovoltaic (PV) properties*,* It refers to the ability of a photovoltaic device to efficiently convert incident sunlight into useable electrical energy [[56], [57], [58]]. As stated, before increased in the number of oligomers increases the LHE value such that 3 – Corannulene and 4-Corannulene had the LHE values of 0.041eV and 0.464 eV respectively. It is important to know that the light harvesting efficiency directly impacts the overall energy conversion efficiency of the device. Higher light harvesting efficiency ensures that a larger fraction of incident sunlight is effectively captured and converted into useable electricity [59].

**Fig. 9:** The process of LHE and Radiative lifetimes (τ) changes in each of the designed structures.

**The open circuit voltage (***V*_**OC**_**):** The open circuit voltage (VOC) stands as a foundational parameter in photovoltaic (PV) systems, symbolizing the peak voltage attainable from a solar cell or module when devoid of any current flow [[60], [61], [62]]. This crucial characteristic offers valuable insights into the photovoltaic properties and performance of the device under study. Equation (13) facilitated the calculation of the open circuit voltage for this research endeavor.

(13) $$V_{OC}=\frac{E_{CB}+\Delta CB}{q}+\frac{kT}{q}In\left(\frac{n_{c}}{N_{CB}}\right)-\frac{E_{Redox}}{q}$$

In accordance with equation (13), the following parameters are defined: ECB denotes the conduction band edge of TiO2, q represents the unit charge, T stands for the absolute temperature, k denotes the Boltzmann constant, nc represents the number of electrons in the conduction band, NCB signifies the density of accessible states in the conduction band, and Eredox represents the redox potential of the electrolyte [[63], [64], [65]]. Additionally, the shift of CB resulting from dye adsorption is mathematically represented by ΔCB in equation (14).

(14) $$\Delta CB=\frac{{q\mu }_{normal}\gamma }{\varepsilon_{0}\epsilon }$$

VOC plays a critical role in determining the energy conversion efficiency of a solar cell or module. It represents the maximum achievable voltage from the solar device, making it a pivotal factor in determining the overall power output. A higher VOC typically indicates a more efficient device. The calculated VOC values for this study were 3.12, 2.37, 2.08, and 1.44 eV, respectively. It is observed that a dye with a smaller energy band gap is advantageous for achieving a red-shifted absorption spectrum, resulting in an increase in the number of electrons (nc) and, consequently, enhancing the device's efficiency. It is noteworthy that the experimental value of ECB employed for the TiO2 semiconductor in this present work was −4.00 eV. This information is crucial for understanding the behavior and performance of the solar cell or module under investigation.

## 4 Conclusions

Advanced theory approaches DFT/CAM-B3LYP and M062X/6-311+G were used in this research to develop and compute the structural, electronic, and optical characteristics of n-Corannulene oligomers (n = 1–4). Corannulene is a molecule composed of fused benzene rings arranged in a bowl-like shape. The number of Corannulene units in a system can significantly impact its electrical conductivity and its relevance for photovoltaic (solar cell) applications. It is worth noting that as the number of Corannulene molecules increases, so does the estimated value of the cohesive energy and the larger the number of units, the greater the potential for extended conjugation and improved charge transport within the material. This property shows Corannulene's proclivity to polymerize to form oligomers. The findings of both calculations indicate that increasing the number of n-Corannulene oligomers increases the HOMO energy while decreasing the LUMO energy. As a result, the energy gap in 4-Corannulene is decreased by 49.5 %. The findings indicated that as the number of oligomers increased, correspondingly increased the dipole moment and the spatial expanse of the electron. Based on the optical activity statistics, it is clear that 4-Corannulene has higher optical activity than other compounds. This structure exhibits one significant absorption in the visible region, suggesting that it is more optically active than the other structures. In reality, increasing the amount of Corannulene units enhanced the optical properties considerably. Moreover, the impacts of the external electric field (EF) on the length of these molecular systems (n-Corannulene) confirmed that the length of each structure diminishes as the intensity of the electric field increases. The relaxation energy for the 4-Corannulene compound was 2.2700 eV, with the highest wavelength of 546.18 nm and oscillator strength of 0.2710 originating from the 200 -> 201(H - > L) orbitals, with a commensurate significant input of (93.33 %).

## Ethics approval and consent to participate

Not applicable.

## Consent for publication

Not applicable.

## Availability of data and material

All data are contained within the manuscript.

## Funding

This research was not funded by any Governmental or Non-governmental agency.

## Authors’ contributions

**Hamid Hadi:** Conceived and designed the experiments. **Terkumbur E. Gber:** Performed the experiments. **Hitler Louis**: Contributed reagents, materials, analysis tools or data, **Festus Ogungbemiro:** Wrote the paper, analyzed and interpreted the data.

## Declaration of competing interest

The authors declare that they have no known competing financial interests or personal relationships that could have appeared to influence the work reported in this paper.
